# Anomalous Behavior Detection Framework Using HTM-Based Semantic Folding Technique

**DOI:** 10.1155/2021/5585238

**Published:** 2021-03-16

**Authors:** Hamid Masood Khan, Fazal Masud Khan, Aurangzeb Khan, Muhammad Zubair Asghar, Daniyal M. Alghazzawi

**Affiliations:** ^1^Institute of Computing and Information Technology, Gomal University, D.I.Khan, Pakistan; ^2^Department of Computer Science, University of Science and Technology, Bannu, Pakistan; ^3^Information Systems Department, Faculty of Computing and Information Technology, King Abdulaziz University, Jeddah, Saudi Arabia

## Abstract

Upon the working principles of the human neocortex, the Hierarchical Temporal Memory model has been developed which is a proposed theoretical framework for sequence learning. Both categorical and numerical types of data are handled by HTM. Semantic Folding Theory (SFT) is based on HTM to represent a data stream for processing in the form of sparse distributed representation (SDR). For natural language perception and production, SFT delivers a solid structural background for semantic evidence description to the fundamentals of the semantic foundation during the phase of language learning. Anomalies are the patterns from data streams that do not follow the expected behavior. Any stream of data patterns could have a number of anomaly types. In a data stream, a single pattern or combination of closely related patterns that diverges and deviates from standard, normal, or expected is called a static (spatial) anomaly. A temporal anomaly is a set of unexpected changes between patterns. When a change first appears, this is recorded as an anomaly. If this change looks a number of times, then it is set to a “new normal” and terminated as an anomaly. An HTM system detects the anomaly, and due to continuous learning nature, it quickly learns when they become the new normal. A robust anomalous behavior detection framework using HTM-based SFT for improving decision-making (SDR-ABDF/P2) is a proposed framework or model in this research. The researcher claims that the proposed model would be able to learn the order of several variables continuously in temporal sequences by using an unsupervised learning rule.

## 1. Introduction

Nowadays, anomalous behavior detection in streaming applications is a challenging task. The system must process data and then output a decision in real time for a quick decision, rather than making many passes or batches of files. Usually in a number of cases of real-world scenarios, the sample of sensor streams is huge enough having a little opportunity for a let alone expert's intervention. Operating in an unsupervised, automated fashion is often a necessity, and as part, the detector should continue to learn and adapt to changing statistics while simultaneously making predictions. Most of the time, the real goal emphasis is prevention, rather than detection, so it is vitally desired and required to detect anomalous behavior as early as possible, giving enough actionable information ideally well before any chance of system failure. It is a difficult task to detect anomalous behavior and compare it with any existing standard. Moreover, in addition to this, real-time applications impose their own specific requirements and challenges that must be considered before taking decisions on results.

### 1.1. Need of Anomalous Behavior Detection

Anomalies are well defined as data patterns that do not conform to expected behavior [1]. A data stream containing different patterns could have several types of anomalies. Spatial (static) anomaly in some cases is a single pattern or can be a set of relatively closely spaced patterns in a data stream that deviates from standard, normal, or expected. A temporal anomaly is a set of surprising transitions between patterns [2, 3]. It is very difficult, and in many cases, it is impossible to detect spatial and temporal anomalies, if the patterns in a data stream are highly random and abrupt. However, it is possible to detect a change in the distribution of the random data, denoted as distribution anomaly [4, 5]. These types of anomalies are named as temporary anomalies. At first when a unique change appears, then it is an anomaly. If it appears a number of times, then it is called “new normal” or behavioral change not to be an anomaly [6].

### 1.2. Research Study Motivation

Hierarchical Temporal Memory (HTM) is a learning system that continuously learns online from the environment [7–9]; it detects temporary anomalies and immediately transforms them when they are the new normal. Input data for HTM functionality is of both types, numerical and categorical. Both data types can be merged in an input data stream to HTM because both are converted to a sparse distributed representation (SDR) using encoders. Each time, HTM calculates an anomaly score for a new pattern as it enters [10–13]. If a received pattern is symmetrical to predict, then the anomaly score is zero. If the pattern is quite different, then the score is one. A partially predicted pattern has a score between zero and one. The SDR of the input data stream determines the similarity. The “similarity” between the actual received pattern and the predicted pattern is the base of HTM score. The larger the overlap between actual and predicted input patterns results in minimal or makes the anomaly score smaller.

HTM learning uses the bursting process at the start. Bursting occurs if none of the cells (bits) in a column were predicted; then, all the cells are made active. It occurs when there is no context. At each time instance, the anomaly score is calculated simply the fraction given by the number of bursting columns divided by the total number of active columns. In the beginning of the training, the anomaly score will be high because most patterns will be new. As HTM learns, the anomaly score will diminish until there is a change in the pattern stream.

### 1.3. Problem Formulation

Keeping in view the HTM model, the main research problem is formulated as follows:

How can we develop a robust framework that can detect anomalous behavior from real-time data streams (microblogs) and convert them into simultaneous prediction vectors based on computed threshold value for comparison using HTM based semantic folding?

### 1.4. Research Contributions

- A robust anomalous behavior detection framework using HTM based on SFT for improving decision making (SDR-ABDF/P2) is proposed
- The proposed model is able to learn order of several variables continuously in temporal sequences by using an unsupervised learning rule
- The proposed technique is also tested on Yelp dataset, and the results were amazingly remarkable. It worked up to showing 96% accuracy
- A number of experiments on different dataset samples have been performed implementing this model successfully
- NAB (Numenta Anomaly Benchmark) is another benchmark that attempts to provide a controlled and repeatable environment of tools to test and measure different anomaly detection algorithms on streaming data

The rest of the article is organized as follows: Section 2 overviews the basic concepts used in this work; in Section 3, we present a review of literature; Section 4 describes proposed methodology; in Section 5, results are analyzed and discussed, and finally, Section 5 focuses on conclusions and future work.

## 2. Preliminary Concepts

The evolution of new technologies for machine intelligence is the discovery of the working principles of neocortex.

### 2.1. Neocortex

The neocortex is not the75% of the brain. Neocortex uses a very common learning algorithm in vision, hearing, touch, behavior, and for everything that has been discovered 35 years ago [14]. Neocortex is an organ of memory that learns through sensory organs like retina, cochlear, and somatic. They form similar matching patterns of actions on cortex [2, 15–17]. The neocortex learns predictive model from continuously variating sensory data. Model generates predictions, anomalies, and action (behavior). Most of the sensory changes are due to movement in sensory organs. The neocortex learns a sensory-motor-model from around the world. The neocortex is the base of intellectual thought in the mammalian brain. Vision, touch, hearing, language, movement, and planning of high level are all performed by the neocortex [18–20]. Given such a diverse collection of cognitive functions, it could be expected that the neocortex to contrivance is an equally diverse suite of specialized neural algorithms. This is not the case. The neocortex displays a remarkably undeviating pattern of neural circuitry [21, 22]. The biological evidence suggests that the neocortex implements a very common set of algorithms to perform many different intelligence functions. Cortical learning algorithm is unbelievably and enormously adoptable in a number of fields like languages, engineering, science, and art. It provides a set of principles. However, a cortical learning algorithm does not provide the best solution to any problem but a generic and flexible solution [23–25]. People like universal solutions to the problems, and nothing is more universal than the human cortex.

### 2.2. Hierarchical Temporal Memory

HTM is an acronym for Hierarchical Temporal Memory, a term used to describe models of neocortex [14]. HTM is a machine learning technology that is aimed at capturing the structural and algorithmic properties of the neocortex [8]. HTM provides only a theoretical framework for understanding the neocortex and its many capabilities [26]. HTMs can be viewed as a type of neural network. However, on its own, the term “neural network” is not very useful because it has been applied to a large variety of systems [27]. HTMs model neurons (in HTM models, they are called cells), which are arranged in columns, in layers, in regions, and in a hierarchy [28].

As the name implies, HTM is basically a memory-based system. HTM networks are trained on a number of time-varying data and depend on storing a large set of patterns and sequences. The data is stored, and retrieved is logically a different way from the standard model used by programmers today. Existing computer memory has a flat organization and does not have an inherent notion and concept of time. A programmer can implement any kind of data organization and structure on top of the flat computer memory. They have control over how and where information is stored [29]. By contrast, HTM memory is more restrictive. HTM memory has a hierarchical organization and is inherently time based. Information is always stored in a distributed fashion. A user of an HTM specifies the size of the hierarchy and what to train the system on, but the HTM controls where and how information is stored [30].

HTM networks are much more different than classic computing; it can be used for general purpose computers to model these HTMs as long as they unified the key functions of hierarchy, time, and sparse-distributed representations. Specialized hardware will be created to generate purpose-built HTM networks [29, 31].

More often, it is illustrated with HTM properties and principles using examples drawn from human vision, touch, hearing, language, and behavior. Such examples are useful because they are intuitive and easily grasped. However, it is important to keep in mind that HTM capabilities are general. They can just as easily be exposed to nonhuman sensory input streams, such as radar and infrared, or to purely informational input streams such as financial market data, weather data, Web traffic patterns, or text. HTMs are learning and prediction machines that can be applied to many types of problems [14].

### 2.3. Semantic Folding Technique

On the basis of HTM, SDRs or semantic folding technique for data-encoding mechanism [32, 33] are used with the following properties:

- Many bits are used to represent a data item, maybe in thousands. Each bit means a neuron (called cell). At a certain point, active is represented by 1, while inactive neurons are represented by 0's
- Few of them are 1's, and most are 0's. For example, within 2000 bits, only 2% are active. Sparsity means that most of the neurons are inactive thus represented by 0's
- Each bit has some meaning known as semantic meaning. Each bit represents a specific feature
- Meaning is learned in this representation. Commonly top forty attributes are taken to represent data

A basic difference between HTM sequence memory and preceding biologically inspired sequence learning models is the use of SDR models [34]. In the neocortex, information is primarily represented by robust activation of a small set of neurons at any time, known as sparse coding [21, 35]. Commonly, HTM sequence memory uses SDRs to represent temporal sequences. Based on mathematical properties of SDRs [26, 32], each neuron (called cell) in the HTM sequence memory model can robustly learn and classify a large number of patterns under unusual and noisy conditions [13]. An ironic distributed neural representation for temporal sequences evolves from computation in HTM sequence memory. Although it is focused on sequence prediction, this representation is valuable for a number of tasks, such as anomaly detection [36] and sequence classification.

Use of a flexible coding scheme is important for online streaming data analytics, where the number of unique symbols is often not known. So more often, it is desired to be able to change the range of the coding scheme at run time without affecting previous learning. This requires a flexible algorithm to use a flexible coding scheme that can represent a large number of unique symbols or a wide range of data [13]. The SDRs used in HTM have a very large coding capacity and allow instantaneous representations of multiple predictions with minimal collisions. These properties make SDR an ideal coding format for the next generation of neural network models [37, 38].

## 3. A Review of Literature

An anomaly is defined as a point in a certain specific time where the performance of the system is unfamiliar and noticeably changed from previous performance. According to this explanation, it is not necessary that an anomaly infers a problem.

### 3.1. Prior Works

Though the use of HTM model using semantic folding technique is the latest model for anomalous behavior detection, however the anomalies in streaming data are heavily studied through years [14]. The founder Subutai Ahmad and Scott Prudy have worked upon the HTM model. In time-series data, anomaly detection is a heavily studied since 1972 [6]. Both supervised and semisupervised methods were used for classification. Though labelled data gives improved results, supervised methods are inappropriate for anomalous behavior detection [11]. Continuous learning which in our case is the requirement is impossible with commonly studied supervised or semisupervised learning algorithms. Other ways, like calculating threshold values, making data clusters, and exponential smoothing, could only be used for spatial anomaly detection [39]. Holt-Winters forecasting as commonly implemented for commercial applications is an example of the latter [40]. Most commonly used are the change point detection methods capable for the identification of temporal anomalies. Another model method is to frame out the time series data in two independent moving windows, and the change is detected as significant deviation in the time series metrics [41, 42]. The computation in these methods is more often enormously fast and has low memory requirements. The anomaly detection performance of statistical methods always remained dependent on the size of e windows and threshold values. With the change in data, the results are turned down due to false positive values and so require updates and changes in threshold values to minimize false positives as to detect anomalies. With the combination of different statistical algorithms, the Skyline project provides an open source implementation of several statistical techniques for detecting anomalies in streaming data [39]. The anomaly detection problem has also been widely studied in the computer security literature where machine learning approach, creating user profiles based on command sequences, compares current input sequences to the profile using a similarity measure. The system learns to classify current behavior as consistent or anomalous with past behavior [43]. Anomalous behavior detection in crowded scenes in the field of computer vision (data streaming) was evaluated on benchmark datasets containing various situations with human crowds, and the results demonstrate that the proposed approach best state-of-the-art methods [44]. A number of other algorithms are used in complex scenarios for the detection of temporal anomalies. For detecting anomalies, ARIMA is a general-purpose method for modeling temporal data (with regular patterns) with seasonality [45], when data occurs in regular patterns. Many extensions have been developed to overcome the problem of seasonality period determination [46]. An improved technique of ARIMA application to multivariate dataset to detect anomaly has also been deeply studied [5]. For segmentation in time series data for online anomaly detection, an approach named Bayesian change point detection method is used [47, 48].EGADS is an open source framework released by Yahoo for anomaly detection that combines common anomaly detection algorithms with time series forecasting techniques [49]. Another open source anomaly detection algorithm for time series data has been released by Twitter [50]. There have been several model-based approaches applied to specific domains, for example, in aircraft engine measurements, anomaly detection method [2], temperature variations in cloud datacenter [3], and detection of frauds in ATM [51]. A few of the other thorough reviews are [1, 52, 53]. But here, our focus is on using HTM for anomalous behavior detection. Derived from working principles of neocortex, a machine learning algorithm HTM has the tendency to model spatial and temporal patterns in continuous streams of data [38, 54]. In sequence prediction, HTM compares to complex non-Markovian sequences [34, 55]. HTMs are continuously learning models that absorb changing statistics automatically, which is a property appropriate to streaming data analysis. Another recent approach for anomalous behavior was made on the dataset of NAB to test the LGMAD algorithm using Long Short-Term Memory and Gaussian Mixture Model [56] with achieving remarkable accuracy.

### 3.2. Research Gap Based on the Limitations of the Previous Studies

A robust anomalous behavior detection framework using HTM based on SFT for improving decision-making (SDR-ABDF/P2) is required, which is what we address in this study. The model should be able to learn order of several variables continuously in temporal sequences by using an unsupervised learning rule.

## 4. Proposed Methodology

The real-time data stream of domain-dependent reviews or microblogs (from yelp dataset) was sent to encoders for converting the data into SDR's representation. These SDRs are applied to HTM model. HTM algorithms work and detect any anomalous behavior in the input data stream from domain-dependent microblogs or reviews.

Proposed methodology is named as SDR-based semantic folding technique based on HTM theory (SDR-ABD/P2) as shown in Figure 1.

SDRs of text inputs are generated, and our proposed method learns behavior from a given text and detects it as an anomaly or not an anomaly. If a text is identified as anomaly, i.e., its behavior is different from already existing texts, the learning process will update itself from this anomaly to set the behavior for next coming inputs (texts). If next text T2 behaves normally, it means the proposed system has learned from previous detected anomaly; otherwise, given text will be excluded from this cluster.

### 4.1. HTM Model Implementation

Sparse distributed representations are the binary vectors designed for the operation of HTM model. These vectors named as SDR provide inputs to HTM. To convert a scalar value of natural language words into binary vectors with a minimum of “active” bits, encoders are used. These SDRs are combined through a pooling process resulting in a semantic space having two percent active bits in a vector of 2048 bits [14]. The HTM model uses a symmetrical model set of parameters for all the experiments.

### 4.2. Encoding

With the help of online carpus, word chunks are encoded into SDR. The encoder creates representations that overlap for inputs that are similar in one or more of the characteristics of the data.

### 4.3. Pooling

It is a temporary space which stores synonyms (obtained from WordNet used as carpus) of all words from all texts without duplicating words. Here, pooler updating and synonym extraction process are both iterative due to the nature of each text having multiple chunks and each chunk having multiple synonyms.

### 4.4. SDR

It is a binary vector where the first row represents the bucket of synonyms for the first text and the second row represents a bucket of synonyms for the second one and so on, and the nth row represents a bucket of synonyms for the nth text. Each row is a list for each text. Each word points to the index of its synonym in pooling/pooler. Learning process is based on the analogy of each coming SDR and will be the union with the previous union-list.

### 4.5. Mathematical Model

(1) Let the vector **Y**_**t**_ represents the state of an input in the form of encoded SDR from real-time microblog system at a certain instantaneous time **t**. A continuous data stream of inputs is exposed to our model
  (1) $$\begin{array}{c} \cdots ..\cdots .Y_{t-2},Y_{t-1},Y_{t},Y_{t+1},Y_{t+2},\cdots \cdots \cdots .. \end{array}$$
(2) In a certain time **t** at each point, it is to know the behavior of the system, either usual or unusual. This determination must be done in real time before time **t** + 1 and without any look ahead. HTM which is a machine learning algorithm tries to match this condition in real time. Since HTM networks are continuously learning and absorb the spatiotemporal features of the inputs
If an input **Y**_**t**_ is given to the system, then the vector **Z**(**Y**_**t**_) is the representation of sparse binary code of input **Y**_**t**_ in time **t**.
  (2) $$\begin{array}{c} Y_{t}=Z\;\left(Y_{t}\right). \end{array}$$
(3) **π**(**Y**_**t**_) is a vector representing a prediction vector for an input **Z**(**Y**_**t**+1_), i.e., a prediction of the next input **Y**_**t**+1_
  (3) $$\begin{array}{c} \pi \left(Y_{t}\right)=Z\left(Y_{t+1}\right). \end{array}$$
(4) Compute the difference and deviation between model's predicted input and the actual input and label as raw anomaly score. The intersection between actual and predicted sparse vectors was the method used to compute. At time **t**, the raw anomaly score is labelled as **S**_**t**_
  (4) $$\begin{array}{c} S_{t}=\pi \left(Y_{t}\right)\cap Z\left(Y_{t+1}\right), \end{array}$$
  and it could therefore be as
  (5) $$\begin{array}{c} s_{t}=1-\frac{\pi \left(Y_{t-1}\right)\cdot Z\left(Yt\right)}{\left|Z\left(Y_{t}\right)\right|}\cdots \cdots \cdots . \end{array}$$
If the prediction of the model is correct and the precisely predicted vector is the same as of the input vector, then raw anomaly score will be 0, else it will be 1 if completely opposite or different. And if the value of **S**_**t**_ lies in between zero and one, it shows the similarity between the input and the prediction vectors.
(5) Based on the HTM model's prediction history, the anomaly likelihood is the only value that defines “how anomalous the current state is”.

If **π**(**Y**_**t**_) is taken as a union of an individual prediction, then the HTM model helps to represent multiple predictions. As the binary vectors are sparse enough with extended dimensionality, with exceptional error chances, a number of predictions can be represented simultaneously as in Bloom filters [39, 57].

### 4.6. Raw Anomaly Score Calculation

Raw anomaly score is the measure needed for calculation of deviation between actual and predicted output at a certain time. It is computed from the intersection between the predicted and actual sparse vectors. For the computation of anomaly likelihood value, a window of the last **W** raw anomaly scores is maintained. The HTM system models this distribution as a rolling normal distribution.

(6) $$\begin{array}{c} W=\sum S_{t}\text{ where }t=1,2,3,4,\cdots \cdots ., \end{array}$$

where sample mean and variance are continuously calculated and updated from previous anomaly scores. As shown under [39],

(7) $$\begin{array}{c} \mu_{t}=\frac{\sum_{i=0}^{i=w-1}s_{t-i}}{k},\\ \delta_{t}^{2}=\frac{\sum_{i=0}^{i=w-1}{\left(s_{t-i}-\mu_{t}\right)}^{2}}{k-1}. \end{array}$$

The distribution is modeled as a rolling normal distribution with the continuous updation of mean and variance from previous anomaly scores. And then an average of recent anomaly scores is computed and applied a threshold to the Gaussian tail probability (Q-function, [58]) to make a decision about declaration of an anomaly. We used this likelihood value as the complement of the tail probability [39].

(8) $$\begin{array}{c} L_{t}=1-Q\left(\frac{\mu \prime_{t}-\mu_{t}}{\delta_{t}}\right), \end{array}$$

where

(9) $$\begin{array}{c} \mu \prime_{t}=\frac{\sum_{i=0}^{i=w-1}s_{t-i}}{j}. \end{array}$$

Anomalous behavior will be reported if **L**_**t**_ > = 1.

*W*′ represents short-term moving average window, where *W*′<<*W*.

SDR-ABDF/P2 thresholds **L**_**t**_ and describes it as detected anomaly if it is very close to 1.

(10) $$\begin{array}{c} \text{Anomaly detected}\equiv L_{t}\geq 1-\varepsilon . \end{array}$$

If **π**(**Y**_**t**_) is taken as a union of an individual prediction, then the HTM model helps to represent multiple predictions. As the binary vectors are sparse enough with extended dimensionality, with exceptional error chances, a number of predictions can be represented simultaneously as in Bloom filters [39, 57].

## 5. Results and Discussion

We had a set of texts named as t1 to t8, where t1, t2, and t3 belong to the same cluster and the text t4 was kept as a partial anomaly. Proposed system learned from t4 and did not detect t5 as a partial anomaly because the system has already updated it from previous inputs. Next, t6 is a partial anomaly, and the system will not be updated according to the new input, i.e., t6, so it will be considered as a pure anomaly. Texts are shown in Table 1.

### 5.1. Pooling Process Application

Table 2 shows an input vector for the pooling process using WordNet, where 1^st^ column contains the synonyms of all chunks in t1, the second column contains the synonyms of all chunks in t2, the third column contains the synonyms of all chunks in t3, and so on.

Table 3 illustrates pooling format where all words from Table 2 are indexed in a way that duplicated words are removed. Hence, 57 words have been indexed from 0 to 56.

### 5.2. SDR Generation

Table 4 shows eight columns, comprising analysis of eight texts. In the 1^st^ column, value [1, ‘big,' 0] narrates synonyms of word “big” in t1 present on “0” index in pooler and so on. All columns are based on the same analogy.

Afterward, an SDR vector is generated from all texts, i.e., row one of SDR for t1 is obtained from column 1 of Table 4, by extracting the last value from each cell showing [“0,” “1,” “1,” “2,” “1,” “1,” “1,” “0,” “3,” “4,” “4,” “5,” “6,” “5”]. Such SDRs for all texts are shown in Table 5.

### 5.3. Anomalous Behavior Detection and Learning Process

It is supposed that in the beginning, the brain of proposed work is empty, and t1 comprises target text, to whom the proposed system will detect similar texts and will learn from new coming text (in data stream). Here, learning is done by making a union of given text with previously detected union, keeping in view that in start union is empty, so t1 will be considered as part of cluster (see Table 6) and then union this text with previous union as shown in the following table.

Now by intersecting the SDR of t2 with the previous union, the elements for t2 are determined. As the number of elements is 5, and in the proposed system, the threshold value is set to 5, so t2 will be considered as similar, i.e., normal text as shown in Table 7. Now from the SDR of t2, the new union is updated.

By repeating the process again, the elements from the intersection of SDR of t3 with previous union, the obtained number of elements is 8, so t3 is considered as similar, i.e., normal text as shown in Table 8. Later on, the new union is updated, from SDR of t3.

Again, by determining the elements from intersection of SDR of t4 with previous union, as these elements are 0, so t4 is considered as partial anomaly text as shown in Table 9 and then updated the new union from SDR of t4.

If succeeding text is not considered as partial anomaly, then t4 will not be a pure anomaly. Now by determining the elements from intersection of SDR of t5 with previous union, the number of obtained elements is 5, so t5 will be considered as similar, i.e., normal text as shown in Table 10, so t4 is not a pure anomaly and updated the new union from SDR of t5.

Determining the elements from intersection of SDR of t6 with previous union, the number of obtained elements is 0, so t6 will be considered as partial anomaly text as shown in Table 11. Again, the new union is updated from SDR of t6.

Similarly, with the elements from intersection of SDR of t7 with previous union, the number of obtained elements is 0, so t7 will be considered as partial anomaly text as shown in Table 12, so t6 is a pure anomaly instead of partial anomaly. Hence, the new union is updated from SDR of t7.

In the last step, by determining the elements from intersection of SDR of t8 with previous union, the total number of elements is 20, so t8 will be considered as normal text as shown in Table 13. And again, new union is updated from SDR of t8.

Precisely, from the above process, it is concluded that t1, t2, t3, t5, and t8 have similar behavior, but t4 is partial anomaly because again t5 has shown normal behavior. Hence, t6 has been considered as pure anomaly because t7 has proved itself as a partial anomaly due to the reason that t8 again is a normal text as shown in Figure 2.

As in our case, the total number of texts is 8, and we have considered the threshold value equal to 5, i.e., (8/2) + 1.

We have detected these anomalies based on different values but found less accurate results. At values 6 and 7, it is found that t2, t4, t5, t6, and t7 are anomalies which are shown in Figure 3.

Although SDR-ABDF/P2 uses HTM as the underlying temporal model, the likelihood technique is not specific to HTMs. It could be used with any other algorithm that outputs a sparse code or scalar anomaly score. The overall quality of the detector will be dependent on the ability of the underlying model to represent the domain.

### 5.4. Statistical Analysis

#### 5.4.1. Data Source

Data has been collected from Yelp dataset (publically available set or reviews) for research. Approximately one hundred and fifty thousand reviews were thought enough for testing and validating our anomalous behavior detection framework named as SDR_ABDF/P2. The collected reviews are converted to SDRs. A sample listing of the said datasets is presented in Table 14 showing three columns of predicted and actual values with the assumptions.

*Actual Category*: “BC” represents behavioral change while “A” represents anomaly, and the numerical value assigned to BC is “1” and to A is “0,”

*True Behavior Change* (*FBC*): If our proposed system determines the value of a review as “1” and the actual value is also “1,” this means it is TBC.

*False Behavior Change* (*TBC*): If our proposed system determines the value of a review as “1” and the actual value is “0,” this means it is FBC.

*True Anomaly* (*TA*): If our proposed system determines the value of a review as “0” and the actual value is also “0,” this means it is TA.

*False Anomaly* (*FA*): If our proposed system determines the value of a review as “0” and the actual value is “1,” this means it is FA.

#### 5.4.2. Confusion Matrix Measures

In machine learning and specifically in statistical classification, a confusion matrix, also called as an error matrix, is a specific table that allows visualization of the performance of an algorithm in supervised learning, while in unsupervised learning, it is called matching matrix. Each row of the matrix represents the instances in a predicted class while each column represents the instances in an actual class or vice versa [59]. It is clear from the name of matrix that confusion matrix makes it easy to see if the system is confusing two classes (i.e., commonly mislabeling one as another). It is also defined as special kind of likelihood table, with two dimensions, one is the “actual” and the other is “predicted,” and identical sets of “classes” in both dimensions [60]. If in any experiment we have “P” positive and “N” negative instances for any condition, the formulated four outcomes 2 × 2*confusion matrix* could be as follows [61, 62].

(11) $$\begin{array}{c} \text{Precision}=\frac{\text{TBC}}{\text{TBC}+\text{FBC},},\\ \text{Recall}=\frac{\text{TBC}}{\text{TBC}+\text{FA}},\\ F-\text{measure}=\frac{2*\text{precision}*\text{recall}}{\text{precision}+\text{recall}}. \end{array}$$

After analysis from the confusion matrix, proposed methodology achieved 96% accuracy and remaining measures are shown in Table 15.

The graphical representation of the results of the sample from yelp dataset is shown in Figure 4:

## 6. Conclusion and Future Work

### 6.1. Conclusion

Upon the working principles of the human neocortex, the HTM model has been developed by Jeff Hawkins, which is a proposed theoretical framework for sequence learning. Both types of data numerical and categorical are best suited input types for HTM model working. SFT is based on HTM to represent a data stream for processing in the form of sparse distributed representation (SDR). SFT offers a framework for unfolding how semantic information is manipulated for natural language observation and creation, towards the details of semantic foundations during the initial language learning phase.

All data patterns that differ from expectation based on previous inputs are called. These anomalies can be of different types. A single data pattern or set of closely spaced patterns when deviated from its normal behavior is called spatial (static) anomaly. When some surprising change occurs between patterns then it is a temporal anomaly. Whenever a sudden change is recorded, it is an anomaly, but when this change appears a number of times, then it is called new normal. Due to continuous learning nature, an HTM primarily detects an anomaly and then quickly transforms into a new normal if the change persists continuously.

A robust anomalous behavior detection framework using HTM based on SFT for improving decision-making (SDR-ABDF/P2) is a proposed framework or model in this research. The researcher claims that the proposed model is able to learn order of several variables continuously in temporal sequences by using an unsupervised learning rule. The proposed technique is also tested on Yelp dataset, and the results were amazingly remarkable. It worked up to showing 96% accuracy. A number of experiments on different dataset samples have been performed implementing this model successfully. NAB (Numenta Anomaly Benchmark) is another benchmark that attempts to provide a controlled and repeatable environment of tools to test and measure different anomaly detection algorithms on streaming data.

### 6.2. Future Suggestions

1. Whenever language models are used in traditional natural language processing with semantic context, proposed system SDR_ABDF/P2 can be used
2. Numeric measurement interpretation as semantic entities is the other area of active research like words. Such research would use log files of historic measurements instead of semantic grounding by reference texts. Measurements of correlation will follow system specific dependencies
3. The next and best area of research is development of hardware architecture. This will uplift the speed of the similarity computation process. In very large semantic search systems holding billions of documents, the bottleneck is the similarity computation. With the use of content addressable memory (CAM) mechanism, the search-by-semantics similarity-process will accelerate at very high velocities

## Figures and Tables

**Figure 1:** Detailed diagram for anomalous behavior detection.

**Figure 2:** Detected anomalies at threshold value 5.

**Figure 3:** Detected anomalies at confidence values 6 and 7.

**Figure 4:** Represents the difference between actual and predicted dataset sample.

**Algorithm 1:** Pseudocode/Algorithm of the Proposed System.

**Table 1:** Samples for dataset.

Texts	Contexts
t1	“big damaged”
t2	“damaged fire”
t3	“fire hot”
t4	“yellow truck.”
t5	“truck silver.”
t6	“too rain”
t7	“happy day”
t8	“fire yellow”

**Table 2:** Input generated vector for pooling.

t1	t2	t3	t4	t5	t6	t7	t8
Large	Damage	Fire	Yellow	Truck	Excessively	Happy	Fire
Big	Damage	Fire	Yellowness	Motor truck	Overly	Felicitous	Fire
Big	Damaged	Firing	Yellow	Hand_truck	To_a_fault	Happy	Firing
Bad	Discredited	Fire	Yellow	Truck	Too	Glad	Fire
Big	Damaged	Flame	Yellowish	Truck	Besides	Happy	Flame
Big		Flaming	Xanthous		Too	Happy	Flaming
Big	Fire	Fire	Chicken	Silver	Also	Well-chosen	Fire
Large	Fire	Fire	Chickenhearted	Ag	Likewise		Fire
Prominent	Firing		Lily-livered	Atomic_number_47	As_well	Day	
	Fire	Hot	White-livered	Silver		Twenty-four_hours	Yellow
Damage	Flame	Hot	Yellow	Ash_grey	Rain	Twenty-four_hour_period	Yellowness
Damage	Flaming	Raging	Yellow-bellied	Ash_gray	Rainfall	24-hour_interval	Yellow
Damaged	Fire	Hot		Silver	Rain	Solar_day	Yellow
Discredited	Fire	Hot	Truck	Silver_grey	Rainwater	Mean_solar_day	Yellowish
Damaged		Blistering	Motortruck	Silver_gray	Rain	Day	Xanthous

**Table 3:** Pooling format for proposed work.

Index	Word	Index	Word
0	Large	29	Atomic_number_47
1	Big	30	Ash_grey
2	Bad	31	Ash_gray
3	Prominent	32	Silver_grey
4	Damage	33	Silver_gray
5	Damaged	34	Excessively
6	Discredited	35	Overly
7	Fire	36	To_a_fault
8	Firing	37	Too
9	Flame	38	Besides
10	Flaming	39	Also
11	Hot	40	Likewise
12	Raging	41	As_well
13	Blistering	42	Rain
14	Red-hot	43	Rainfall
15	Yellow	44	Rainwater
16	Yellowness	45	Pelting
17	Yellowish	46	Rain_down
18	Xanthous	47	Happy
19	Chicken	48	Felicitous
20	Chickenhearted	49	Glad
21	Lily-livered	50	Well-chosen
22	White-livered	51	Day
23	Yellow-bellied	52	Twenty-four_hours
24	Truck	53	Twenty-four_hour_period
25	Motortruck	54	24-hour_interval
26	Hand_truck	55	Solar_day
27	Silver	56	Mean_solar_day
28	Ag		

**Table 4:** Generated input from pooling for SDR.

t1	t2	t3	t4	t5	t6	t7	t8
[1, “big,” 0]	[2, “damaged,” 4]	[3, “fire,” 7]	[4, “yellow,” 15]	[5, “truck,” 24]	[6, “too,” 34]	[7, “silver,” 27]	[8, “fire,” 7]
[1, “big,” 1]	[2, “damaged,” 4]	[3, “fire,” 7]	[4, “yellow,” 16]	[5, “truck,” 25]	[6, “too,” 35]	[7, “silver,” 28]	[8, “fire,” 7]
[1, “big,” 1]	[2, “damaged,” 5]	[3, “fire,” 8]	[4, “yellow,” 15]	[5, “truck,” 26]	[6, “too,” 36]	[7, “silver,” 29]	[8, “fire,” 8]
[1, “big,” 2]	[2, “damaged,” 6]	[3, “fire,” 7]	[4, “yellow,” 15]	[5, “truck,” 24]	[6, “too,” 37]	[7, “silver,” 27]	[8, “fire,” 7]
[1, “big,” 1]	[2, “damaged,” 5]	[3, “fire,” 9]	[4, “yellow,” 17]	[5, “truck,” 24]	[6, “too,” 38]	[7, “silver,” 30]	[8, “fire,” 9]
[1, “big,” 1]	[2, “fire,” 7]	[3, “fire,” 10]	[4, “yellow,” 18]	[5, “silver,” 27]	[6, “too,” 37]	[7, “silver,” 31]	[8, “fire,” 10]
[1, “big,” 1]	[2, “fire,” 7]	[3, “fire,” 7]	[4, “yellow,” 19]	[5, “silver,” 28]	[6, “too,” 39]	[7, “silver,” 27]	[8, “fire,” 7]
[1, “big,” 0]	[2, “fire,” 8]	[3, “fire,” 7]	[4, “yellow,” 20]	[5, “silver,” 29]	[6, “too,” 40]	[7, “silver,” 32]	[8, “fire,” 7]
[1, “big,” 3]	[2, “fire,” 7]	[3, “hot,” 11]	[4, “yellow,” 21]	[5, “silver,” 27]	[6, “too,” 41]	[7, “silver,” 33]	[8, “yellow,” 15]
[1, “damaged,” 4]	[2, “fire,” 9]	[3, “hot,” 11]	[4, “yellow,” 22]	[5, “silver,” 30]	[6, “rain,” 42]	[7, “damaged,” 4]	[8, “yellow,” 16]
[1, “damaged,” 4]	[2, “fire,” 10]	[3, “hot,” 12]	[4, “yellow,” 15]	[5, “silver,” 31]	[6, “rain,” 43]	[7, “damaged,” 4]	[8, “yellow,” 15]
[1, “damaged,” 5]	[2, “fire,” 7]	[3, “hot,” 11]	[4, “yellow,” 23]	[5, “silver,” 27]	[6, “rain,” 42]	[7, “damaged,” 5]	[8, “yellow,” 15]
[1, “damaged,” 6]	[2, “fire,” 7]	[3, “hot,” 11]	[4, “truck,” 24]	[5, “silver,” 32]	[6, “rain,” 44]	[7, “damaged,” 6]	[8, “yellow,” 17]
[1, “damaged,” 5]		[3, “hot,” 11]	[4, “truck,” 25]	[5, “silver,” 33]	[6, “rain,” 42]	[7, “damaged,” 5]	[8, “yellow,” 18]
		[3, “hot,” 11]	[4, “truck,” 26]		[6, “rain,” 45]		[8, “yellow,” 19]
		[3, “hot,” 13]	[4, “truck,” 24]		[6, “rain,” 42]		[8, “yellow,” 20]
		[3, “hot,” 11]	[4, “truck,” 24]		[6, “rain,” 46]		[8, “yellow,” 21]
		[3, “hot,” 14]					[8, “yellow,” 22]
							[8, “yellow,” 15]
							[8, “yellow,” 23]

**Table 5:** SDR for all texts.

Texts	SDR
t1	[“0,” “1,” “1,” “2,” “1,” “1,” “1,” “0,” “3,” “4,” “4,” “5,” “6,” “5”]
t2	[“4,” “4,” “5,” “6,” “5,” “7,” “7,” “8,” “7,” “9,” “10,” “7,” “7”]
t3	[“7,” “7,” “8,” “7,” “9,” “10,” “7,” “7,” “11,” “11,” “12,” “11,” “11,” “11,” “11,” “13,” “11,” “14”]
t4	[“15,” “16,” “15,” “15,” “17,”, “18” “19,” “20,” “21,” “22,” “15,” “23,” “24,” “25,” “26,” “24,” “24”]
t5	[“24,” “25,” “26,” “24,” “24,” “27,” “28,” “29,” “27,” “30,” “31,” “27,” “32,” “33”]
t6	[“34,” “35,” “36,” “37,” “38,” “37,” “39,” “40,” “41,” “42,” “43,” “42,” “44,” “42,” “45,” “42,” “46”]
t7	[“47,” “48,” “47,” “49,” “47,” “47”, “50”, “51”, “52”, “53”, “54”, “55”, “56”, “51”, “51”]
t8	[“7,” “7,” “8,” “7,” “9,” “10,” “7,” “7,” “15,” “16,” “15,” “15,” “17,” “18,” “19,” “20,” “21,” “22,” “15,” “23”]

**Table 6:** Becoming t1 as part of cluster.

Previous union	Empty
	-----
Set of t1	[“0,” “1,” “1,” “2,” “1,” “1,” “1,” “0,” “3,” “4,” “4,” “5,” “6,” “5”]

**Table 7:** Inserting t2 as part of cluster.

(Updated learning process) union with t1	0 1 2 3 4 5 6
Set of t2	[“4,” “4,” “5,” “6,” “5,” “7,” “7,” “8,” “7,” “9,” “10,” “7,” “7”]
	t2: with previous union: common words 5

**Table 8:** Inserting t3 as part of cluster.

Union with t2	0 1 2 3 4 5 6 7 8 9 10
Set of t3	[“7,” “7,” “8,” “7,” “9,” “10,” “7,” “7,” “11,” “11,” “12,” “11,” “11,” “11,” “11,” “13,” “11,” “14”]
	t3: with previous union: common words 8

**Table 9:** Partial anomaly t4.

Union with t3	0 1 2 3 4 5 6 7 8 9 10 11 12 13 14
Set of t4	[“15,” “16,” “15,” “15,” “17,” “18,” “19,” “20,” “21,” “22,” “15,” “23,” “24,” “25,” “26,” “24,” “24”]
	t4: with previous union: common words 0

**Table 10:** Inserting t5 as part of cluster.

Union with t4	0 1 2 3 4 5 6 7 8 9 10 11 12 13 14 15 16 17 18 19 20 21 22 23 24 25 26
Set of t5	[“24,” “25,” “26,” “24,” “24,” “27,” “28,” “29,” “27,” “30,” “31,” “27,” “32,” “33”]
	t5: with previous union: common words 5

**Table 11:** Partial anomaly t6.

Union with t5	0 1 2 3 4 5 6 7 8 9 10 11 12 13 14 15 16 17 18 19 20 21 22 23 24 25 26 27 28 29 30 31 32 33
Set of t6	[“34,” “35,” “36,” “37,” “38,” “37,” “39,” “40,” “41,” “42,” “43,” “42,” “44,” “42,” “45,” “42,” “46”]
	t6: with previous union: common words 0

**Table 12:** Partial anomaly t7 and pure anomaly t6.

Union with t6	0 1 2 3 4 5 6 7 8 9 10 11 12 13 14 15 16 17 18 19 20 21 22 23 24 25 26 27 28 29 30 31 32 33 34 35 36 37 38 39 40 41 42 43 44 45 46
Set of t7	[“47,” “48,” “47,” “49,” “47,” “47,” “50,” “51,” “52,” “53,” “54,” “55,” “56,” “51,” “51”]
	t7: with previous union: common words 0

**Table 13:** Becoming t8 as part of cluster.

Union with t7	0 1 2 3 4 5 6 7 8 9 10 11 12 13 14 15 16 17 18 19 20 21 22 23 24 25 26 27 28 29 30 31 32 33 34 35 36 37 38 39 40 41 42 43 44 45 46 47 48 49 50 51 52 53 54 55 56
Set of t8	[“7,” “7,” “8,” “7,” “9,” “10,” “7,” “7,” “15,” “16,” “15,” “15,” “17,” “18,” “19,” “20,” “21,” “22,” “15,” “23”]
	t8: with previous union: common words 20

**Table 14:** A sample from Yelp dataset as processed.

S.no	Text	Predicted	Actual category	Actual
1	“Wow loved this place”	1	BC	1
2	“Crust is not good”	0	A	0
3	“It is not tasty and the texture was just nasty”	1	BC	1
4	“Stopped by during the late may bank holiday off Rick Steve recommendation and loved it”	1	A	0
5	“The selection on the menu was great and so were the prices”	1	BC	1
6	“Now I am getting angry and I want my damn pho”	1	BC	1
7	“Honestly, it did not taste that fresh”	1	BC	1
8	“The potatoes were not fresh and like rubber and you could tell they had been made up ahead of time being kept under a warmer”	1	BC	1
9	“The fries were great too”	1	BC	1
10	“A good great touch”	1	BC	1
11	“Service was very prompt”	1	BC	1
12	“Would not go back”	1	BC	1
13	“The cashier had no care whatsoever on what I had to say it still ended up being way overpriced”	1	A	0
14	“I tried the cape cod ravoli”	1	BC	1
15	“I was disgusted because I was pretty sure that was human hair”	1	BC	1
16	“I was shocked because no signs indicate cash only”	1	A	0
17	“Highly demanded”	0	A	0
18	“Waitress was a little slow in service”	1	BC	1
19	“This place is not worth your time”	1	BC	1
20	“Did not like at all”	1	BC	1

**Table 15:** Showing precision and recall for both categories.

Category	Precision	Recall	f1-score
0	1.00	0.60	0.75
1	0.96	1.00	0.98
Average	0.96	0.96	0.96

## Data Availability

Underlying data supporting the results can be provided by sending a request to the corresponding author.
